The article "Using mathematical models to evaluate germination rate and seedlings length of chickpea seed (Cicer arietinum L.) to osmotic stress at cardinal temperatures" was retracted in 2022. Reasons: compromised peer review; a conflict of interest; concerns about the authorship.

# Using mathematical models to evaluate germination rate and seedlings length of chickpea seed (*Cicer arietinum* L.) to osmotic stress at cardinal temperatures

**DOI:** 10.1371/journal.pone.0260990

**Published:** 2021-12-17

**Authors:** Sikandar Shah, Sami Ullah, Sajjad Ali, Ajmal Khan, Muhammad Ali, Said Hassan

**Affiliations:** 1 Department of Botany, University of Peshawar, Peshawar, Khyber Pakhtunkhwa, Pakistan; 2 Department of Botany, Bacha Khan University, Charsadda, Khyber Pakhtunkhwa, Pakistan; 3 Institute of Biotechnology and Microbiology, Bacha Khan University, Charsadda, Khyber Pakhtunkhwa, Pakistan; The University of Haripur, PAKISTAN

## Abstract

*Cicer arietinum* is the 3^rd^ most important cool season legume crop growing in vast arid and semi-arid regions of the world. A lab experiment was designed using hydrothermal time model (HTT) to investigate the chickpea seed germination (SG) behavior, cardinal temperatures and germination responses across fluctuating temperatures (*T*_s_) and water potentials (*Ψ*_s_). Seeds of chickpea var. NIFA 1995 were germinated at six constant *T*_s_ (7, 14, 21, 28, 35 and 42°C) each having the following five water potentials: 0, -0.2, -0.4–0.6 and -0.8 MPa. Germination percentage (G%) decreased significantly at (*P ≤ 0.05) from 86.7% at 28°C in -0.2 MPa to 10% in -0.2 MPa at 7°C. The germination rate (GR = 1/t_50_) against different *T* percentiles exhibited that linear increase was observed in the GR pattern above and below the *T*_o._ Based on the confidence intervals of the model coefficients and (*R*^*2*^: 0.96), the average cardinal temperatures were 4.7, 23 and 44.2°C for the base (*T*_b_), optimal (*T*_o_) and ceiling (*T*_c_) temperatures respectively. *θT*1 value was observed maximum at 28°C in -0.2 MPa and decreases with decreasing *Ψ* (-0.8 MPa). In comparison with control, the *θT*2 value was also highest in -0.2 MPa at 28°C. The thermal time (TT) concept is well fitted to germination fraction data in distilled water with an *R*^*2*^ value increasing 0.972. The hydro time constant (*θ*H) increased with an increase in *T* to *T*_o_ and then decreased when *T*>*T*_o_. The *ѱ*_b(50)_ irregularly varied with increasing *T*, σ*Ψ*_b_ was also recorded lowest (0.166 MPa) at 28°C and highest (0.457 MPa) at 7°C. Based on the statistical analysis, cardinal temperatures, hydrothermal time constant (*θ*HTT) and germination findings the HTT gives an insight into the interactive effect of *T* and *Ψ* on seed germination time courses under varying environmental conditions.

## 1. Introduction

Chickpea (*Cicer arietinum* L.) is the 3^rd^ most authoritative cool season grain legume crop after the *Phaseolus vulgaris* and *Pisum sativum*, which are grown in vast arid and semi-arid regions of the world [1]. It is documented as one of the famous and oldest pulses cultivated from ancient times both in Europe and in Asia. Chickpea seeds are a decisive and inexpensive source of highly digestible nutrients such as vitamins, proteins, carbohydrates, minerals and potentially health beneficial phytochemicals especially for people in underprivileged countries [2]. After Turkey and India, Pakistan is the third largest commercial producer of chickpeas with a 7% segment in global production [3, 4]. In Pakistan, chickpea covers 73% of the land and shares 76% of the gross production [5, 6]. SG is the first and most complex morphological and physiological phase in the succession of plant development where many factors such as temperature, water potential, drought and flood affect it [7]. Temperature (*T*) and water potential (*Ψ*) are the two most important external features that affect seed germination rate and germination characteristics [8]. Depending on the water potential of the permeation medium, if it is reduced germination may be also stopped or decelerated [9]. GR is correlated with the differential magnitude between environment water potential and physiological threshold water potential for the emergence of seed radicle [10]. Similarly, when water is not limited, the soil temperature is the most important environmental factor affecting seed germination and consequently plant establishment in the field [11].

The earth’s climate is changing drastically in recent decades and these climate changes affect all the physiological phases of plant growth and development [12]. This changing climate increases the intensity and frequency of the abiotic factors that contrarily reduced agricultural production [13]. In these abiotic factors, temperature is the key factor affecting seed germination parameters in all plants [14]. However, it is significant that each taxon requires a certain range of *T*s for seed germination called cardinal temperatures [15]. These are the minimum or base temperature (*T*_b_), maximum or ceiling temperature (*T*_c_) at which germination rate is minimum and optimum temperature (*T*_o_) at which maximum germination occurs in a short period [16].

Gummerson developed mathematical thermal time (TT), hydro time (HT) and hydrothermal time model (HTT) to study the eco-physiological responses of seed germination to *T*, *Ψ* and their interaction (*T* × *Ψ*) [17]. Models can be quite useful in forecasting seed emergence time, dormancy and its use in crop management. Seed germination in the TT model is summarized in three cardinal temperatures (base, ceiling and optimum temperature). Similarly, the HT model is also described in three parameters (**a**) base water potential (*Ψ*_b_) (**b**) hydro time constant (*θ*H) and (**c**) Standard deviation of the base water potential (σ*Ψ*_b_) [10]. The base water potential is the theoretical threshold describing the prevention of seed germination fraction. TT, HT and HTT are the best models for describing seed germination patterns with *T*, *Ψ* and their interactions (*T* × *Ψ*). In recent times, the hydrothermal time model has been extensively used by many researchers to individually and simultaneously inspect the results of both *T* and *Ψ* on seed germination outlines in several plants such as safflower (*Carthamus tinctorius* L.) [18], carrot (*Daucus carota*) [19], watermelon (*Citrullus vulgaris*) [20] as well as in weedy species.

Therefore, the objective of the current research work was: (**i**) to inspect the SG of *C*. *arietinum* at several *T*_s_, *Ψ*_s_ and their interactions (*T* × *Ψ*) (**ii**) to explain chickpea seed SG behavior using models of the thermal time, hydro time and hydrothermal time (**iii**) to determine SG cardinal *T*_s_ and drought tolerance threshold (base water potential). To the best of our knowledge, this is the first research study from Pakistan related to the application of the HTT model to predict the germination patterns of *C*. *arietinum* under various *T*_s_ and *Ψ*_s_.

## 2. Materials and methods

### 2.1. Seeds description and experiment protocol

Chickpea (*Cicer arietinum* L.) var. NIFA 1995 seeds were brought from Nuclear Institute for Food and Agriculture (NIFA), Peshawar, Khyber Pakhtunkhwa, Pakistan with a 95% viability rate. The variety is described as light brown, angular shaped with an average weight (0.22±2gm) and length (0.4±1cm). Before the experiment, the seeds were stored in sealed plastic bags at 4°C in dark.

The seeds were surface sterilized with 95% ethanol solution for 3 minutes and then washed with distilled water and shade dried at room temperature. The experiment was conducted according to randomized complete block design (RCBD), at various *Ψ*_s_ and *T*_s_ in an incubator (Memmert Beschickung-Loading-Model 100–800, Germany) from October to December 2020 at Plant Physiology Lab. Department of Botany, University of Peshawar [5, 21]. The experiment comprised of a wide range of constant temperatures (7, 14, 21, 28, 35 and 42°C) each having the following four *Ψ*s (distilled water), -0.2, -0.4–0.6 and -0.8 MPa. The polyethylene glycol (PEG6000; Merck, Germany) was used for the preparation of *Ψ*_s_ solutions as suggested by [22]. Five accelerated aging periods (APP) of 24, 48, 72, 96 and 120 hours were used.

The standard germination test was performed by placing 35 seeds on Wathman No. 1 filter paper in Petri dishes moistened with 5 ml distilled water and PEG6000 solutions. The Petri dishes were randomly placed in an incubator in dark except for reading times. Each treatment has three replicates. Seeds were considered to have germinated when the radicle was 1 mm in length and was observed each day. The experiment was completed after 120 hours and germinated seeds were removed and counted for their germination parameters.

### 2.2. Data analysis

The germination data was analyzed through repeated probit regression analysis defined by [23, 24] which is based on TT, HT and HTT models. The germination rate (GR) was calculated as the inverse of the germination time for each percentile at each *T* or *Ψ*.

### 2.3. Thermal time (TT)

The germination time course data of constant *T*_*s*_ at each *Ψ* was quantified through the thermal time (TT) concept.

At sub-optimal *T*s the model was:

θT1=TTsub=(T–Tb)t Eq (1)

and at supra-optimal *T*s the model was:

θT2=TTsupra=(Tc(g)−T)tg Eq (2)

Hence the germination rate is the reverse of the seed emergence time, the Eqs (1) and (2) can be written as Eq (3):

GR=1/tg=(T−Tb(g))/θT Eq (3)

Where *θT*1 and *θT*2 are the thermal time constant, *T* is the actual temperature of germination, *T*_b_ is the base temperature for germination fraction, g is the actual time to germination fraction, GR_(g)_ is the germination rate of the seed population.

### 2.4. Hydro time (HT)

Modeling of SG in response to *Ψ*_s_ and accelerated aging period was analyzed using the hydro time model as suggested by [17]. *θ*H determines the relationships between solute potential and germination rate in the same way as the thermal time model. The model can be expressed as:

$$\theta H_{\left(g\right)}=(\psi -\psi b)tg$$ Eq (4)

$$GR_{\left(g\right)}=1/tg=\psi -\psi b)/\theta H$$ Eq (5)

Where *θ*H is the hydro time constant (MPa.h), *Ψ* is actual water potential, *Ψ*_b(g)_ is the base water potential of germination fraction g (%), tg is the time of seed population for radicle emergence, GR_(g)_ is the germination rate is the actual time to germination fraction g. These parameters can be used as an indicator to evaluate seed vigor and quality in a seed lot.

### 2.5. Hydrothermal time model (HTT)

The TT and HT models can be combined into a joint hydrothermal time model to predict and describe the SG patterns in response to varied *T* and *Ψ* in a single seedbed. In terms of the HTT model, the germination time course at all *T*_s_ and *Ψ* in the sub-optimal *T* (from *T*_b_ to *T*_o_) can be described as:

θHTT=(Ψ–Ψb(g))(T−Tb)tg Eq (6)

θHTT=[Ψ–Ψb(g)–(kT(T–To))](T–Tb)tg Eq (7)

Where *θ*HTT is the hydrothermal time constant (MPa h) that has a constant value of seed population. *T*_o_ is the predicted optimum temperature for germination fraction. k_T_ is Boltzmann constant (slope of C_b(g)_ versus *T* when *T*>*T*_o_).

### 2.6. Germination attributes

The following germination indices were calculated from the per day and cumulative germination, physical observation, radicle and plumule lengths and fresh and dry weight of the seedlings.

#### 2.6.1. Germination percentage (G%)

G% represent the total number of seeds germinated out of the total seeds sown in each Petri dish. This germination parameter was calculated from the formula used by Onofri et al. [24].


$$Germination\;Percentage\;(G\%)=\frac{Final\;number\;of\;seedling\;emerged}{Total\;number\;of\;seeds\;sown}\times 100$$ Eq (8)

#### 2.6.2. Germination energy (GE)

Seed germination energy was calculated by using the formula suggested by Thriunavukkarasu and his colleagues [25].


$$Germination\;Energy\;(GE)=\frac{X1}{Y1}+(\frac{X2-X1}{Y2})+(\frac{Xn-Xn-1}{Yn})$$ Eq (9)

#### 2.6.3. Mean germination time (MGT)

The MGT index showed that how fast the seeds emerged in a population. Small MGT value means seed population has a high rate and vice versa. This was calculated by the formula of Onofri et al. [24].


$$Mean\;Germination\;Time\;(MGT)=\frac{\in fx}{\in f}$$ Eq (10)

#### 2.6.4. Coefficient of velocity of germination (CVG)

The CVG represents the velocity of germination of seeds in an experiment. This will increase with an upsurge in the frequency of germinated seeds. The highest theoretical CVG value will be obtained when all sown seeds germinated on the first day. This was calculated from the formula suggested by Shah et al. [12].


$$Coefficient\;of\;Velocity\;of\;Germination\;(CVG)=\frac{N1+N2+N3\ldots Nx}{100}\times N1T1\ldots .NxTx$$ Eq (11)

#### 2.6.5. Germination index (GI)

The Germination index tells us about the germination percentage and speed of germination. GI was calculated from the methodology of Labrie et al. [26].


GerminationIndex(GI)=(10×n1)+(9n×n2)…(1n×10) Eq (12)

#### 2.6.6. Germination rate index (GRI)

The GRI represent the percent germination on respective day and time. It was calculated by using the method of Rashidi [27].


$$Germination\;Rate\;Index\;(GRI)=\frac{G1}{1}+\frac{G2}{2}+\frac{G3}{3}\ldots .\frac{Gx}{x}$$ Eq (13)

#### 2.6.7. Seed vigor index-1 (SVI-1)

The length of three seedlings from each pot was measured in cm and then calculated by using the formula suggested by Chen et al. [28].


SeedVigorIndex(SVI‐1)=Seedlingslength(cm)×SeedGermination%age Eq (14)

#### 2.6.8. Seed vigor index-II (SVI-II)

The dry weight of three seedlings from each pot was determined through electrical balance and then multiply with seed germination percentage as suggested by Chen et al. [28].


SeedVigorIndex‐II(SVI‐II)=Seedlingdryweight×Germintion%age Eq (15)

#### 2.6.9. Time to 50% germination (T50%)

This index was developed to find out the time required for 50% seed germination. T50% was calculated through a mathematical formula developed by Hao et al. [29].


$$Time\;to\;50\%\;Germination\;(T50\%)=\frac{ti+(N/2-ni)(tj-ti)}{\left(nj-ni\right)}$$ Eq (16)

#### 2.6.10. Timson germination index (TGI)

The TGI index represents the average number of seeds germinated per day. This was measured according to the method of Hao et al. [29].


$$Timson\;Germination\;Index\;(TGI)=\frac{\in G}{T}$$ Eq (17)

### 2.7. Data analysis

The investigation of *T*_s_ (thermal time), *Ψ*_s_ (hydro time) and their interactions (hydrothermal time model) on seed germination rate and germination attributes were analyzed through linear regression using IBM SPSS Statistics 26 and SigmaPlot Version 11.0. The basic statistical calculation was performed in excel software (S1 File). The values of the following parameters: *ѱ*_b(50),_ σ*Ψ*_b_; *R*^*2*^, SE, Sig, F and T-test were determined using linear probit regression analysis in SPSS. ORIGIN 2021 PC Corporation was used for plotting various graphs of germination fraction vs accelerated aging period and germination parameters against *T* and *Ψ*.

## 3. Results

### 3.1. Germination responses to fluctuating temperatures (TT model)

Initially, the increase in temperature amplitude endorsed germination rate and percentage of seeds but decreased as *T* exceeds certain limit. Table 1 showed that temperature had significant (*P≤0.05) effects on germination rate (GR = 1/t_50_) and percentage of *Cicer arietinum* var NIFA-1995. Under optimum moisture (0 MPa) the highest G% was recorded at 28°C and lowest at 7 and 42°C (Fig 1A and 1F). In general, the minimum germination (10 and 16.3%) was reported at 7 and 42°C under -0.8 MPa and maximum (86.7%) at 28°C under -0.2 MPa in comparison with control (Fig 1A and 1F). It means germination increased from 40% to 93.3% with increasing temperature up to 28°C, then decreased again to 40% as the temperature exceeds from 28°C (optimum *T*) to 42°C. In general germination percentage increased with AAP and significantly (*P≤0.05) decreased with high *T* (Fig 1A–1F). According to the results a substantially high *θ*T1 value was observed at 28°C in -0.2 MPa and decreases with decreasing *Ψ* (-0.8 MPa) irrespective of species investigated (Table 1). In comparison with control, *θ*T2 value was also documented highest in (-0.2 MPa) at 28°C. The TT concept is well fitted to germination fraction data in distilled water with *R*^*2*^ value increasing 0.972 (Table 2). Plotting the germination rate against different *T* percentiles exhibited that linear increase was observed in GR_(g)_ pattern above and below the *T*_o_ (Table 1)_._ Using the same pattern but in opposite direction, the GR_(g)_ values showed significant (**P≤0.01) increment with decreasing *Ψ* (more negative) at all *Ts*. The base water potential at 50 percentile (*ѱ*_b(50)_) showed an irregular pattern with increasing temperature. Similarly, the F and T-test also showed a lop-sided behavior having no linear pattern, except that both values were recorded maximum at 28°C (Table 2). Initially, these GR_(g)_ responses are applied to compute the base, optimum and ceiling temperature values.

**Fig 1:** Cumulative germination fraction for *Cicer arietinum* at (**a**) 7°C, (**b**) 14°C, (**c**) 21°C, (**d**)28°C, (**e**)35°C and (**f**) 42°C having different water potentials (0, -0.2, -0.4, -0.6, -0.8 MPa). Symbols indicate water potential and lines indicate cumulative germination fraction predicted by hydrothermal time model.

**Table 1:** The estimated parameters of the hydro and thermal time model to describe *Hordeum vulgare* L. seed germination under different temperatures (*T*s) and water potentials (*ѱs*).

T	Ψ (MPa)	TTsub (θT1)	TTsupra (θT2)	θH (MPa h)	θHTT (MPa h)	Hydro time GR_(g)_	Thermal time GR_(g)_
15°C	0	768	1920	38.4	384	0.013	0.013
	-0.5	544	1360	27.2	272	0.018	0.018
	-1.0	448	1120	22.4	224	0.022	0.022
	-1.5	448	1120	22.4	224	0.022	0.022
	-2.0	96.0	240.0	4.8	48.0	0.104	0.104
20°C	0	896	2240	44.8	448	0.011	0.011
	-0.5	736	1840	36.8	368	0.014	0.014
	-1.0	640	1600	32.0	320	0.016	0.016
	-1.5	448	1120	22.4	224	0.022	0.022
	-2.0	128	320.0	6.40	64.0	0.078	0.078
25°C	0	640	1600	32.0	320	0.016	0.016
	-0.5	448	1120	22.4	224	0.022	0.022
	-1.0	320	800.0	16.0	160	0.031	0.031
	-1.5	320	800.0	16.0	160	0.031	0.031
	-2.0	96.0	240.0	4.80	48.0	0.104	0.104
30°C	0	576	1440	28.8	288	0.017	0.017
	-0.5	448	1120	22.4	224	0.022	0.022
	-1.0	352	880.0	17.6	176	0.028	0.028
	-1.5	224	560.0	11.2	112	0.045	0.045
	-2.0	96.0	240.0	4.80	48.0	0.104	0.104
35°C	0	256	640.0	12.8	128	0.039	0.039
	-0.5	416	1040	20.8	208	0.024	0.024
	-1.0	320	800.0	16.0	160	0.031	0.031
	-1.5	320	800.0	16.0	160	0.031	0.031
	-2.0	96.0	240.0	4.80	48.0	0.104	0.104
40°C	0	224	560.0	11.2	112	0.045	0.045
	-0.5	96.0	240.0	4.80	48.0	0.104	0.104
	-1.0	96.0	240.0	4.80	48.0	0.104	0.104
	-1.5	64.0	160.0	3.20	32.0	0.156	0.156
	-2.0	32.0	80.0	1.60	16.0	0.313	0.313

Temperatures (T); Water potential (ψ); Thermal time constant at sub-optimal temperature (TTsub); Thermal time constant at supra-optimal temperature (TTsupra); Hydrotime constant (*θ*H); Hydrothermal time constant (θHTT); Germination rate (GR).

**Table 2:** Prediction of the hydrotime model parameters for chickpea using non-linear regression at each temperature.

Temperature	*ѱ*_b(50)_ (MPa)	σ*ψ*_b_ (MPa)	*R* ^*2*^	SE	F	T	Sig.
7°C	-0.91	0.457	0.960	1.431	72.00	18.47	0.003^b^
14°C	-0.58	0.328	0.959	1.937	69.81	19.42	0.003^b^
21°C	-1.28	0.174	0.893	3.648	24.92	13.36	0.015^b^
28°C	-1.10	0.166	0.972	2.186	103.7	27.78	0.002^b^
35°C	-1.27	0.290	0.661	6.686	5.860	7.161	0.094^b^
42°C	-0.31	0.201	0.870	1.915	20.16	11.64	0.021^b^

Base water potential at 50 percentile (ѱ_b(50)_); Standard deviation in *Ψ*_b_ (σψ_b_**)**_;_ Coefficient of determination (*R*^*2*^); Standard error (SE); Variability between different means (F); Test (T); Level of significance (Sig).

### 3.2. Germination responses to water potentials (*ѱ*_s_) (HT model)

The variation in seed germination time courses against water potential was scrutinized separately at each *T* (*R*^*2*^ ranges 0.661–0.972) using the hydro time model. *θ*H, *Ψ*, *ѱ*_b_ and GR_(g)_ parameters for our experimental data at each constant *T* and various *ѱ* were analyzed by this HT concept. The minimum G% of 10% was recorded at 7°C in -0.8 MPa and the maximum 86.3% in -0.8 MPa at 28°C (Fig 1A and 1D). Generally, the highest G% was observed in -0.2 MPa and lowest in -0.8 at all *T* (Fig 1A–1F).

It is observed that decreasing osmotic potential of the imbibition solution significantly reduced and delayed germination percentage and this inhibition effect was more severe at a temperature above and below optimum *T*. Both of these values showed minute increment with accelerated aging periods. The highest hydro time constant (*θ*H) (41.6 MPa h) value was recorded in -0.2 MPa at 28°C and lowest at 7°C in -0.8 MPa in comparison with control (Table 1). The data set of *θ*H resulted from water potentials and germination fractions of seed population were plotted against constant *T*. The median base water potential (*ѱ*_b(50)_) values were irregularly varied with increasing temperature having values ranging from -1.28 to -0.58 MPa (Table 2). The standard deviation (σ*Ψ*_b_) of the base water potential at 50 percentiles was also recorded lowest (0.166 MPa) at 28°C and highest (0.457 MPa) at 7°C. The GR_(g)_ of the HT concept showed a remarkable high value at 7°C in -0.8 MPa (Table 2).

### 3.3. Germination responses to temperature and water potential (HTT model)

The seed germination responses to integrating the effect of temperature and water potential above the thermal threshold (*T*_b_) and the hydro threshold (*ѱ*_b_) can be quantified using the hydrothermal time model. The HTT concept predictability was maximum (*R*^*2*^ = 0.960 at 7°C) at suboptimal temperatures (*T***<***T*_o_) than at supra optimal temperature (*R*^*2*^ = 0.872) (Table 2). The interaction of *T* and *Ψ* pointedly affected G% and GR (*P<0.05). The comparative results of the HTT model showed that the effect of water potential on seed germination is slightly high as compared to temperature. The highest hydrothermal time constant (*θ*HTT) value was observed in -0.2 MPa at 28°C as compare to control (0 MPa). A linear pattern of increasing *θ*HTT was followed as *T* increases up to optimal and decreases as we move towards ceiling *T*. Across various water potentials, the *θ*HTT values decrease with decreasing osmotic potential (negative *ѱ*). The estimated cardinal temperatures of the HTT concept were 4.7°C for *T*_b_, *T*_o_ is 23°C and *T*_c_ is 44.2°C respectively in control (Table 3).

**Table 3:** Estimated variable values using the hydrothermal time model for describing seed germination and cardinal temperatures of *Cicer arietinum* L. at six constant *T*s at each of the following four *ψ*s.

Variables		*Cicer arietinum* var. NIFA 1995
**Hydrothermal time model parameters**		
*Ѱ*b (50) (MPa)		-1.34
σ*ψ*b (MPa)		2.65
θHTT (MPa°Ch^-1^)		34.56
kT (MPa°Ch^-1^)		0.104
**Cardinal temperatures**		
*T*_b_ (°C)		4.7
*T*_o_ (°C)		23
*T*_c_ (°C)		44.2
*R* ^*2*^		0.96

Boltzmann constant *(*kT); Coefficient of determination (*R*^2^), Base temperature (*T*_b_); Optimum temperature (*T*_o_); Ceiling temperature (*T*_c_).

Data of the germination attributes were presented in 3D graphs plotted against *T* and *ѱ*. Statistical analysis and graphical presentation revealed a significant change at (*P≤0.05) in radicle length, plumule length, G%, GE, MGT, CVG, GI, GRI, SVI-I and II, TGI and T50% in comparison with control treatment (Figs 2–4). The parameters which were affected negatively by increasing water potential (more negative) and temperature includes radicle length, plumule length, G%, GE, CVG, GI, GRI, SVI-I, SVI-II and TGI (Figs 2A–2D, 3B–3D and 4A–4C). These indices were reported highest in -0.2 MPa at 28°C. On the contrary, the parameters MGT and T50% were reported maximum in -0.8 MPa at 42°C (Figs 3A and 4D). The increasing pattern in these two indices is opposite with osmotic potential and temperature in comparison with above.

**Fig 2:** Interactive effect of water potential and temperature on (A) Radicle length (B) Plumule length (C) Germination percentage (D) Germination energy of chickpea var. NIFA 1995.

**Fig 3:** Interactive effect of water potential and temperature on (**A**) Mean germination time (**B**) Coefficient of velocity of germination (**C**) Germination energy (**D**) Germination rate index of chickpea var. NIFA 1995.

**Fig 4:** Interactive effect of water potential and temperature on (**A**) Seed vigor index-I (**B**) Seed vigor index-II (**C**) Timson germination index (**D**) Time to 50% germination of chickpea var. NIFA 1995.

## 4. Discussion

Finding a suitable geographic location, where a species can germinate and be established successfully, required studying germination patterns under the influence of various abiotic factors. In this aspect mathematical model (TT, HT and HTT model) aids to determine and quantify the effect of these abiotic factors on seed germination time courses in seed lot [30]. Among these abiotic factors, *T* is one of the devastating stress affecting seed germinations in several plants [31, 32]. Stress related to water (*ѱ)* is also major environmental factor limiting early seedling and seed germination [33, 34]. Our results also demonstrated that seed germination was significantly affected by *T* and water stress (*ѱ*).

Our research findings showed that in *Cicer arietinum* G% significantly decreased at a temperature above and below *T*_o_ (28°C) (Fig 2C). The decreased in G% is due to the thermal denaturation of essential amino acids required for seed germination [35]. Similarly, the decreasing pattern of G% continued with decreasing water potential. The highest G% was recorded in -0.2 MPa as compared to control and lowest in -0.8 MPa at all the six constant temperatures (Fig 1A–1F). Decreasing *ѱ* resulted in the consumption of water potential energy and as a result, the supply of water is limited to seed [36]. Our germination findings against *ѱ* can be validated with the studies of [16] and [19] for watermelon and zucchini. The GR_(g)_ showed a linear decreasing correlation with *T* up to *T*_s_≤*T*_o_ at constant *ѱ*, which is in agreement with the TT data on *Hordeum sponataneum* [37]. The *T*_b_ obtained (4.7°C) for chickpea in our experiment is lower than the given *T*_b_ (7°C) (Table 3). The *T*_b_ is an essential cardinal temperature required in developing a crop simulation model and suitable growing time [38]. The *T*_o_ calculated in our study was 23°C which is in agreement with [16]. Generally, seeds are incubated at a constant *T* in the laboratory, but they practice an inclusive range of *T* variations during the emergence time in the field. Seeds under changing *T* accumulated less thermal time than under constant *T* conditions [39]. The *T*_c_ estimated (44.2°C) in our study was probably equal to [40]. Based on the model behavior the cardinal temperature values were unaffected by *ѱ* in our experiment, which inversed with Mesgaran (*Daucus carota*) [39], (*Retama raetam*) [41] and corroborated with Bakhshandeh [8]. The amount *θ*H resulted from water potentials and germination fractions increased with increasing *T* at sub-optimal *T*. The GR_(g)_ values plotted against *T* also showed a slight decline with increasing *T* at constant *ѱ* (Table 1). The *θ*H and GR_(g)_ results are in contrast with the findings of [16] in *Sesamum indicum* and [31] in *Allium tenuissimum*. However, with reducing water potential the GR_(g)_ values increased results of our experiment are in line with the findings of [42] for lemon balm and [20] for watermelon. In research studies and breeding programs, the *θ*H values were used to categorize cultivars and varieties in terms of their sensitivity to *ѱ*.

The values of base water potential at 50 percentiles ѱ_b(50)_ showed an irregular pattern and were minimum (-1.28 MPa) at 21°C and maximum at 42°C (Table 2). Due to thermo-inhibition [20] also reported that *ѱ*_b(50)_ values were minimal at sup optimal *T* and become positive (increasing) at supra optimal *T*. Results indicated that σ*Ψ*_b_ values followed a liner probit trend of decreasing with increasing *T* up to *T*_o_ and then irregular pattern at supra optimal *T*. This can be associated to a reduction in the activity of enzymes and oxygen demand during SG time. The σ*Ψ*_b_ is used as an indicator to represent uniform changes in seed germination in seed lot [43]. However, based on estimated hydro time parameters (*θ*H, *Ψ*_b(50)_ and *σΨ*_b_) we can easily forecast whole germination time courses at any *T* and *Ψ*.

The TT and HT concepts are successfully applied in many types of researches to explain SG behaviors at *T* (sub and supra) and *Ψ*. But the TT concept showed an error at suboptimal *T*_*s*_ by not predicting the decline in GR when *T*_s_>*T*_o_ [30]. As a result, the HTT model was developed by Bradford to overcome the problem [44]. Now the HTT concept is a robust method to study how the interaction of environmental factors (*T* and *Ψ*) influence SG in seed lot [20 and 30]. The hydrothermal time constant (*θ*HTT) estimated for chickpea was 34.56 (MPa°Ch^-1^) (Table 3). Reduction in the seed germination characteristics such as radicle, plumule length, G%, GRI, GI, CVG, GE, SVI-I and II and TGI against high *T* and low *ѱ* have also been reported. High *T* and low *Ψ* cause these reductions due to thermo-inhibition of cellular mechanisms and chemical reactions in the seed [44 and 45]. The influence of these stresses is most prominent in crop agronomy because these attributes signify the component of highest concern to farmers, as well as consumers [46, 47]. Based on the statistical analysis, cardinal temperatures, *θ*HTT and germination findings the HTT give an insight into the interactive effect of *T* and *Ψ* on seed germination populations.

## 5. Conclusions and novelty perspectives

The results of our findings indicated that G% and GR were significantly affected by *T*, *Ψ* and their interactions with accelerated aging periods. The HTT model developed has a clear physiological meaning and characterizes the response of *C*. *arietinum* SG behavior at all *T*_s_ and *Ψ*_s_. The GR and its attributes notably reduced across all the high *T* (35 and 42°C) and reduced *Ψ* (-0.8 MPa). Based on the TT, HT and models the highest *θ*T1 and *θ*T2 values were observed in -0.2 MPa at 28°C, lowest and highest *θ*H values at -0.8 MPa at 7°C and -0.2 MPa at 28°C, for HTT model predicted *θ*HTT average value is 34.56 (MPa°Ch^-1^), *Ѱ*_b(50)_ is -1.34 MPa and σ*Ψ*_b_ value 2.65 MPa at k_T_ 0.104 MPa°Ch^-1^ and cardinal *T*_s_ (*T*_b_ = 4.7°C, *T*_o_ = 23°C and *T*_c_ = 44.2°C. According to available literature, no specific seed germination patterns research has been reported from Pakistan to date for *Cicer arietinum* using the hydrothermal time model. This is the first detailed study on any mathematical model to describe germination patterns of chickpea. While the germination parameters were also described for the first time through our study for chickpea under water stress and temperature. Eventually, the HTT model provides a detailed quantitative description of *C*. *arietinum* SG to develop the physiological status of chickpea seed populations.

## Supporting information

S1 File List of all the statistical calculations and germination indices that were performed in the experiment. (XLSX)

## Abbreviations

T: Temperature
σΨ_b_: Standard deviation of Ψ_b_
Ψ: Water potential
TTsub: Sub optimal temperature
MPa: Megapascal
TTsupra: Supra optimal temperature
T_b_: Base temperature
θH: Hydrotime time constant
T_o_: Optimum temperature
Ψ_b(50)_: The base Ψ of 50^th^ percentile
T_c_: Ceiling temperature
GR: Germination rate or 1/tg
Ψ_b_: Base water potential
G%: Germination percentage
HTT: Hydrothermal time
TT: Thermal time

## References

[1] VermaM, KumarV, PatelRK, GargR, JainM. CTDB: an integrated chickpea transcriptome database for functional and applied genomics. PLoS ONE. 2015; 108: e0136880. doi: 10.1371/journal.pone.0136880 26322998PMC4556341

[2] Mahdavi MashakiK, GargV, Nasrollahnezhad GhomiAA, KudapaH, ChitikineniA, ZaynaliNezhad, et al. RNA-Seq analysis revealed genes associated with drought stress response in kabuli chickpea (*Cicer arietinum* L.). PLoS ONE. 2018; 13(6): e0199774. doi: 10.1371/journal.pone.0199774 29953498PMC6023194

[3] DawarK, FahadS, JahangirMMR, MunirI, AlamSS, KhanSA, et al. Biochar and urease inhibitor mitigate NH_3_ and N2O emissions and improve wheat yield in a urea fertilized alkaline soil. Sci Rep. 2021; 11(1), 1–11. doi: 10.1038/s41598-020-79139-8 34465833PMC8408238

[4] RaniU, SinghS, BasandraiAK, RatheeVK, TripathiK, SinghN, et al. Identification of novel resistant sources for ascochyta blight (*Ascochyta rabiei*) in chickpea. PLoS ONE. 2020; 15(10): e0240589. doi: 10.1371/journal.pone.0240589 33075085PMC7571675

[5] ShahS, KhanS, ShahSM, KhanS, KhatakL, & RukhG. Ethnoecological appraisal, mineral and phytochemical analysis of five species of Myrtaceae in University Campus, Peshawar, Pakistan. Pure and Applied Biology. 2020; 10(1), 244–253. 10.19045/bspab.2021.100025.

[6] YounisU., RahiA. A., DanishS., AliM. A., AhmedN., DattaR., et al. Fourier Transform Infrared Spectroscopy vibrational bands study of *Spinacia oleracea* and *Trigonella corniculata* under biochar amendment in naturally contaminated soil. PLoS ONE. 2020; 16(6), e0253390. 10.1371/journal.pone.0253390.PMC824485234191839

[7] BakhshandehE, GholamhossieniM. Quantification of soybean seed germination response to seed deterioration under peg-induced water stress using hydro time concept. Acta Physiol Planta. 2018; 40(7): 1–8. doi: 10.1007/s11738-018-2700-1

[8] BakhshandehE, HemmatollahP, FatemehV, MobinaG. Quantification of the effect of environmental factors on seed germination and seedling growth of Eruca (*Eruca sativa*) using mathematical models. J Plant Growth Regul. 2020a; 39(1): 190–204. doi: 0.1007/s00344-019-09974-1

[9] MahmoodA, AwanMI, SadafS, MukhtarA, WangX, FiazS, et al. Bio-diesel production of sunflower through sulphur management in a semi-arid subtropical environment. Environ Sci Pollut Res. 2021; 1–11. doi: 10.1007/s11356-021-16688-z 34585347

[10] SaberaliSF, Shirmohamadi-AliakbarkhaniZ, 2020a. Quantifying seed germination response of melon (*Cucumis melo* L.) to temperature and water potential: Thermal time, hydro time and hydrothermal time models. S Afr J Bot. 2020a; 130: 240–249. doi: 10.1016/j.sajb.2019.12.024

[11] PatanèC, SaitaA, TubeilehA, CosentinoSL, CavallaroV. Modeling seed germination of unprimed and primed seeds of sweet sorghum under PEG-induced water stress through the hydro time analysis. Acta Physiol Planta. 2016; 38(5): 1–12. doi: 10.1007/s11738-016-2135-5

[12] ShahW, UllahS, AliS, IdreesM, KhanMN, AliK, et al. Effect of exogenous alpha-tocopherol on physio-biochemical attributes and agronomic performance of lentil (*Lens culinaris* Medik.) under drought stress. PloS ONE. 2021; 16(8): e0248200. doi: 10.1371/journal.pone.0248200 34358230PMC8345888

[13] VaughanMM, BlockA, ChristensenSA, AllenLH, SchmelzEA. The effects of climate change associated abiotic stresses on maize phytochemical defenses. Phytochem Rev. 2018; 17(1): 37–49. doi: 10.1007/s11101-017-9508-2

[14] ShahS, KhanS, SulaimanS, MuhammadM, BadshahL, BussmannRW, et al. Quantitative study on medicinal plants traded in selected herbal markets of Khyber Pakhtunkhwa, Pakistan. Ethnobot. Res. Appl. 2020; 20, 1–36. doi: 10.32859/era

[15] BakhshandehE GholamhossieniM. Modelling the effects of water stress and temperature on seed germination of radish and cantaloupe. J Plant Growth Regul. 2019; 38(4): 1402–1411. doi: 10.1007/s00344-019-09942-9

[16] BaathGS, KakaniVG, GowdaPH, RocateliAC, NorthupBK, SinghH, et al. Guar responses to temperature: Estimation of cardinal temperatures and photosynthetic parameters. Ind Crops Prod. 2020; 145. 111940. doi: 10.7717/peerj.8866 32292650PMC7147430

[17] BakhshandehE, JamaliM, AfshoonE, GholamhossieniM. Using hydrothermal time concept to describe sesame (*Sesamum indicum* L.) seed germination response to temperature and water potential. Acta Physiol Planta. 2017; 39(11); 1–9. doi: 10.1007/s11738-017-2549-8

[18] GummersonRJ. The effect of constant temperatures and osmotic potentials on the germination of sugar beet. J Exp Bot. 1986; 37(6): 729–741. 10.1139/cjb-2015-0166.

[19] BidgolyRO, BalouchiH, SoltaniE, MoradiA. Effect of temperature and water potential on *Carthamus tinctorius* L. seed germination: Quantification of the cardinal temperatures and modeling using hydrothermal time. Ind Crops Prod. 2018; 113, 121–127. doi: 10.1016/J.INDCROP.2018.01.017

[20] AtashiS, BakhshandehE, MehdipourM, JamaliM, Da SilvaJAT. Application of a hydrothermal time seed germination model using the Weibull distribution to describe base water potential in zucchini (*Cucurbita pepo* L.). J Plant Growth Regul. 2015; 34(1): 150–157. 10.1007/s00344-014-9452-y.

[21] BasitA, KhanS, Sulaiman, ShahS, & ShahAA. Morphological features of various selected tree species on the greater university campus Peshawar, Pakistan. Int J Bot Studies. 2019; 4, 92–97. doi: 10.22271/botany/2019

[22] BakhshandehE, AtashiS, HafezniaM, PirdashtiH, da SilvaJAT. Hydrothermal time analysis of watermelon (*Citrullus vulgaris* cv.‘Crimson sweet’) seed germination. Acta Physiol Planta. 2015; 37(1): 1738. doi: 10.1007/s11738-014-1738-y

[23] SanehkooriFH, PirdashtiH, BakhshandehE. Quantifying water stress and temperature effects on camelina (*Camelina sativa* L.) seed germination. Environ Exp Bot. 2021; 186: 104450. 10.1016/j.envexpbot.2021.104450.

[24] OnofriA, BenincasaP, MesgaranMB, RitzC. Hydrothermal-time-to-event models for seed germination. Eur J Agron. 2018; 101: 129–139. s://doi.org/10.1016/j.eja.2018.08.011.

[25] MoltchanovaE, SharifiaminaS, MootDJ, ShayanfarA, BloombergM. Comparison of three different statistical approaches (non-linear least-squares regression, survival analysis and Bayesian inference) in their usefulness for estimating hydrothermal time models of seed germination. Seed Sci Res. 2020; 30(1): 64–72. 10.1017/S0960258520000082.

[26] LabrieG, GagnonAÈ, VanasseA, LatraverseA, TremblayG. Impacts of neonicotinoid seed treatments on soil-dwelling pest populations and agronomic parameters in corn and soybean in Quebec (Canada). PLoS ONE. 2020; 15(2): e0229136. doi: 10.1371/journal.pone.0229136 32101547PMC7043745

[27] ShahS., KhanS., BussmannR. W., AliM., HussainD., & HussainW. Quantitative ethnobotanical study of Indigenous knowledge on medicinal plants used by the tribal communities of Gokand Valley, District Buner, Khyber Pakhtunkhwa, Pakistan. Plants. 2020; 9(8), 1001. doi: 10.3390/plants9081001 32781736PMC7463859

[28] LouY, ZhaoP, WangD, AmomboE, SunX, WangH, et al. Germination, physiological responses and gene expression of tall fescue (*Festuca arundinacea* Schreb.) growing under Pb and Cd. PLoS ONE. 2017; 12(1): e0169495. doi: 10.1371/journal.pone.0169495 28046098PMC5207687

[29] RashidiA, TehranifarA, SamieiL. Improving energy efficiency, germination indices and root system development in Cape periwinkle and marigold through spectral distribution and light exposure time. Environ Exp Bot. 2021; 104531. 10.1016/j.envexpbot.2021.104531.

[30] KhanS, HussainW, ShahS, HussainH, AltyarAE, AshourML, et al. Overcoming Tribal Boundaries: The Biocultural Heritage of Foraging and Cooking Wild Vegetables among Four Pathan Groups in the Gadoon Valley, NW Pakistan. Biology. 2021; 10(6), 537. doi: 10.3390/biology10060537 34203868PMC8232688

[31] HaoJH, LvSS, BhattacharyaS, FuJG. Germination response of four alien congeneric Amaranthus species to environmental factors. PLoS ONE. 2017; 12(1): e0170297. doi: 10.1371/journal.pone.0170297 28107495PMC5249158

[32] XiaoH, YangH, MonacoT, SongQ, RongY. Modeling the influence of temperature and water potential on seed germination of *Allium tenuissimum* L. PeerJ; 2020; 8: e8866. doi: 10.7717/peerj.8866 32292650PMC7147430

[33] WangH, ZhaoK, LiX, ChenX, LiuW, WangJ. Factors affecting seed germination and emergence of *Aegilops tauschii*. Weed Res. 2020; 60: 171–181. 10.1111/wre.12410.

[34] BakhshandehE, BradfordKJ, PirdashtiH, VahabiniaF, AbdellaouiR. A new halothermal time model describes seed germination responses to salinity across both sub-and supra-optimal temperatures. Acta Physiol Planta. 2020b; 42(8): 1–15. 10.1007/s11738-020-03126-9.

[35] WijewardanaC, AlsajriFA, ReddyKR. Soybean seed germination response to in vitro osmotic stress. Seed Technol. 2018; 39: 143–154. https://www.jstor.org/stable/45135884.

[36] DawadiD, SeepaulR, GeorgeS, GrootJ, WrightD. Drought tolerance classification of common oilseed species using seed germination assay. J oil seed Brassica. 2019; 10: 97–105.

[37] MollaeeM, DarbandiEI, AvalMB, ChauhanBS. Germination response of three Setaria species (*S*. *viridis*, *S*. *verticillata*, and *S*. *glauca*) to water potential and temperature using non-linear regression and hydrothermal time models. Acta Physiol Planta. 2020; 42(9): 1–14. doi: 10.1007/s11738-020-03133-w

[38] BradfordKJ. Water relations in seed germination. In Seed development and germination 1995; 351–396 Routledge.

[39] MesgaranMB, OnofriA, MashhadiHR, CousensRD. Water availability shifts the optimal temperatures for seed germination: A modelling approach. Ecol Modell. 2017; 351: 87–95. doi: 10.1016/j.ecolmodel.2017.02.020

[40] LuoT, XianM, KhanMN, HuL, XuZ. Estimation of base temperature for germination of rapeseed (*Brassica napus* L.) using different models. Int J Agric Biol. 2018: 20, 524–530. doi: 10.17957/IJAB/15.0512

[41] SaberaliSF, Nastari NasrabadiH, et al. 2020b. Simulation of Germination Response of Watermelon (*Citrullus lanatus* Thunb.) to Temperature and Water Potential. J Hortic Sci. 2020b; 33(4): 727–741. doi: 10.22067/JHORTS4.V33I4.80628

[42] BakhshandehE, AtashiS, Hafez-NiaM, PirdashtiH. Quantification of the response of germination rate to temperature in sesame (*Sesamum indicum*). Seed Sci Technol. 2013; 41(3): 469–473.

[43] AbdellaouiR, BoughallebF, ZayoudD, NeffatiM, BakhshandehE. Quantification of Retama raetam seed germination response to temperature and water potential using hydrothermal time concept. Environ Exp Bot. 2019; 157: 211–216.

[44] AtashiS, BakhshandehE, ZeinaliZ, YassariE, Teixeira da SilvaJA. Modeling seed germination in *Melissa officinalis* L. in response to temperature and water potential. Acta Physiol Planta. 2014; 36: 605–611. doi: 10.1007/s11738-013-1436-1

[45] BradfordKJ, StillDW. Applications of hydrotime analysis in seed testing. Seed Technology 2004; 75–85. https://www.jstor.org/stable/23433495.

[46] EkinciR, BaşbağS, KarademirE, KarademirÇ. The effects of high temperature stress on some agronomic characters in cotton. Pak J Bot. 2017; 49(2): 503–508. https://hdl.handle.net/20.500.12604/469.

[47] NemeskériE, HelyesL. Physiological responses of selected vegetable crop species to water stress. Agronomy. 2019; 9(8): 447. 10.3390/agronomy9080447.

